# Study of the biological function of LncRNA LUCAT1 on cervical cancer cells by targeting miR-199b-5p

This article has been retracted.

**DOI:** 10.1042/BSR20200422

**Published:** 2020-04-21

**Authors:** Ting Yang, Shengnan Xia

**Affiliations:** Department of Obstetrics, Fourth People’s Hospital of Jinan, Jinan, Shandong Province, China

**Keywords:** cervical cancer, diagnosis, invasion, LUCAT1, miR-199b-5p, proliferation

## Abstract

To explore the effect and mechanism of LncRNA LUCAT1 in cervical cancer (CC). In the present study, 67 cases of CC patients and 60 healthy cases were selected as the research objects. CC patients were selected as the study group (SG) and healthy physical examination patients were selected as the control group (CG). LUCAT1 expression level in peripheral blood was detected in the two groups. Human cervical carcinoma cells C33A, AV3 and normal cervical epithelial cells H8 were purchased for biological behavior analysis. LUCAT1 was highly expressed in SG and cancer tissues (*P*<0.050), and it had good diagnostic value for the development of CC (*P*<0.001). It was closely related to the differentiation, pathological stage and metastasis of CC (*P*<0.001). The prognosis of CC patients was affected (*P*<0.050). After transfecting LUCAT1 into CC cells, it was found that the proliferation, invasion ability and anti-apoptosis protein of CC cells were significantly reduced, while the apoptosis rate and apoptosis protein were significantly increased by inhibiting LUCAT1 expression (*P*<0.050). However, after transfecting miR-199b-5p into CC cells, it was found that the proliferation, invasion ability and anti-apoptosis protein of CC cells were significantly increased, while the apoptosis rate and apoptosis protein were significantly decreased by inhibiting LUCAT1 expression (*P*<0.050). LUCAT1 was highly expressed in CC. It was involved in the tumor development of CC by targeting miR-199b-5p, which was of great significance for the diagnosis and treatment of CC in the future.

## Introduction

Cervical cancer (CC) is a malignant tumor occurring in the uterus and vagina and cervical canal. Currently, it is the most common gynecologic malignant tumor, mostly occurring in the middle-aged and elderly people. In recent years, the incidence rate has shown a significant trend of getting younger [1,2]. According to statistics, the incidence rate of CC has reached 6–29% worldwide at present [3], and approximately 200000 women die of CC every year [4]. At present, surgery or its combination with radiotherapy and chemotherapy is commonly used in clinical treatment of CC, which has a good therapeutic effect for patients with with early stage tumor. However, the cure rate for middle and advanced patients is very low [5,6]. According to previous data, the period of precancerous lesions of CC is relatively long, up to approximately 10 years [7]. At present, the main methods are still surgery or its combination with radiotherapy and chemotherapy for the treatment of CC in clinical practice. For patients with early stage tumor, the effect is still significant, and it can effectively cure CC. For some patients with tumor metastasis or degree of invasion, tumor lesions are usually unable to be completely removed, the prognosis of patients with recurrence is relatively high, and survival is not objective. Therefore, it is of great significance to fully understand the pathogenesis of CC for the prevention and treatment of CC. At present, the pathogenesis of CC is not yet clear. Some researches conclude that early marriage, early pregnancy, prolificacy, sexual disorder and bacteria may be one of the causes of CC [8]. With the deepening of research, more and more researches begin to focus on genetic changes.

LncRNA is a non-coding RNA with a length of more than 200 nucleotides. LncRNA plays an important role in many life activities such as dose compensation effect, epigenetic regulation, cell cycle regulation and cell differentiation regulation. It has been proved to be closely related to many tumor diseases [9,10]. LncRNA LUCAT1 has been proved to be involved in ovarian cancer and thyroid carcinoma [11,12] in previous studies, but its role in CC is still unclear. We speculated that LUCAT1 might be closely related to the occurrence of CC. It may be used as an effective blood marker to improve the detection rate of early CC in the future. Besides, targeted therapy of LUCAT1 can improve the therapeutic effect of CC in clinical practice. In order to verify this point, this experiment aimed to provide new reference ideas for future clinical diagnosis and treatment of CC by exploring the clinical significance and mechanism of LUCAT1 in CC.

## Materials and methods

### Patients’ data

From June 2014 to June 2016, 67 cases of CC patients and 60 healthy cases were selected as the research objects. CC patients were selected as the study group (SG) and healthy physical examination patients were selected as the control group (CG). The present study was approved by the Fourth People’s Hospital of Jinan ethics committees and the present study is in line with the Declaration of Helsinki. All subjects have signed the informed consent. The general data of patients were compared in the two groups. There was no statistical difference in age, BMI, smoking, drinking, marital status, fertility condition, living environment, nationality, etc. (*P*>0.050).

### Inclusion and exclusion criteria

#### Inclusion criteria

Patients conformed to the clinical manifestations of CC and they were diagnosed as CC after biopsy by Pathology Department in the Fourth People’s Hospital. Patients met AJCC TNM staging standard [13]. Patients had complete case data; patients agreed to cooperate and participate in this investigation and experiment. Informed consent was signed by the patient himself or his immediate family members.

#### Exclusion criteria

Patients with multiple tumors were excluded. Patients which received tumor-related treatment within half a year before admission were excluded. Patients with other congenital diseases were excluded. Patients with autoimmune defects were excluded. Patients with liver and renal insufficiency due to organ failure were excluded. Patients with low treatment compliance for mental disorders were excluded. Patients with drug allergy were excluded. Patients who died during treatment were excluded. Patients whose expected survival time was less than 1 month were excluded. Patients who transferred to other hospitals were excluded.

#### Inclusion and exclusion criteria in CG

All subjects were healthy cases in the Fourth People’s Hospital and they had no major medical history. All the results of physical examination were normal. They agreed to cooperate with the investigation.

### Cell data

Human cervical carcinoma cells C33A (BNCC341097), HeLa (BNCC342189), AV3 (BNCC340836) and normal cervical epithelial cells H8 (BNCC340657) were all purchased from BeNa Culture Collection, a subsidiary agency of ATCC. DMEM containing 10% fetal bovine serum (FBS) and 1% penicillin/streptomycin mixture was used to culture in an incubator at 37°C and 5% CO_2_. When the cell grew to approximately 80% fusion degree, trypsin was used to digest for approximately 1 min. The culture medium was used to replaced according to the ratio of 1: 3 and passaged once every 2 days.

### Main instruments and reagents

There was RIPA reagent (Thermo Fisher Scientific, U.S.A., 89901), protein extraction reagent (Thermo Fisher Scientific, U.S.A., 87787), ECL fluorescence kit (Thermo Fisher Scientific, U.S.A., 32209), trypsin (Thermo Fisher Scientific, U.S.A., 25300120), Lipofectamine™ 2000 Transfection Reagent (Thermo Fisher Scientific, U.S.A., 11668019), TransScript II Green Two-Step qRT-PCR SuperMix, TransScript Green miRNA Two-Step qRT-PCR SuperMix (TransGen Biotech, Beijing, AQ301-01, AQ202-01), CCK-8 kit (Shanghai Yisheng Biotechnology Co., LTD., 40203ES60), Transwell kit (Gibco, U.S.A., 1142802), DMEM (Thermo Fisher Scientific, U.S.A., A2493901), PBS (Thermo Fisher Scientific, U.S.A., 20012050), fetal bovine serum (Thermo Fisher Scientific, U.S.A., 10099141C), Penicillin–Streptomycin (Gibco, U.S.A., 15070063), Annexin V/PI apoptosis assay kit (Shanghai Yisheng Biotechnology Co., LTD., 40310ES60), double luciferin reporter gene assay kit (Promega, U.S.A.) and CEZMagna RIP kit (Millipore, Billerica, MA, U.S.A.).

### Detection methods

#### PCR detection

The collected blood sample was extracted with EasyPure miRNA Kit for total RNA. The extracted total RNA was detected for purity, concentration and integrity by ultraviolet spectrophotometer and agarose gel electrophoresis. The 2× TS miRNA Reaction Mix in the TransScript Green miRNA Two-Step qRT-PCR SuperMix kit was used for RNA reverse transcription to cDNA. The specific procedures were performed according to the manufacturer’s kit instructions. Then PCR amplification experiment was carried out. PCR system was as follows: cDNA 1 μl, upstream and downstream primers each 0.4 μl, 20× TransTaq® Tip Green qPCR SuperMix 10 μl, Passive Reference Dye (50×) 0.4 μl. In the end, ddH_2_O was added to complete to 20 μl. PCR conditions were as follows: pre-degeneration at 94°C for 30 s, degeneration at 94°C for 5 s, annealing and extension at at 60°C for 15 s, with a total of 40 cycles. Three repeated wells were set up in each sample. The experiment was carried out three times. LncRNA used U6-1 as internal parameters. miRNA used U6-2 as internal parameters. 2^−△△q*C*_t_^ was used to analyze the data (Table 1).

**Table 1:** Primer sequence

	F (5′–3′)	R (3′–5′)
LUCAT1	AGCTCCACCTCCCGGGTTCACG	CGTGAACCCGGGAGGTGGAGCT
miR-199b-5p	GCCCGCCCAGTGTTTAGAC-TAT	GTGCAGGGTCCGAGGT
U6-1	CTCGCTTCGGCAGCACA	AACGCTTCACGAATTTGCGT
U6-2	CTCGCTTCG-GCAGCAC	AACGCTTCACGAATTT-GCGT

### Cells transfection

The expression level of LUCAT1 was detected in each group of cell lines, and the two with the most significant difference were selected for subsequent transfection experiments. LUCAT1 (si-LUCAT1), overexpression LUCAT1 (sh-LUCAT1) and NC would be knocked down. The sequences of knockdown miR-199b-5p (inhibition-miR-199b-5p), overexpression of miR-199b-5p (mimics-miR-199b-5p) and NC (NC-miR) were transfected into CC cells according to the instructions of liposome Lipofectamine™ 2000. After transfection for 6 h, the medium was changed for routine culture for 48 h. The transfection efficiency was detected by qRT-PCR. After successful transfection, it was used for subsequent tests.

### MTT experiment

Twenty microliters of 5 g/l of MTT solution was added. The supernatant was discarded after culture for 4 h. One hundred fifty microliters of dimethyl sulfoxide (DMSO) was added to each hole and fully shaken to dissolve the crystals. The absorbance (A) of the cells was detected at 490 nm wavelength.

### Flow cytometry

The transfected cells were digested with 0.25% trypsin and washed twice with PBS. One hundred microliters of binding buffer was added to prepare into 1 × 10^6^/ml suspension. AnnexinV-FITC and PI were successively added and incubated at room temperature and in dark for 5 min. FC500MCL flow cytometer system was used for detection. The experiment was repeated for three times to take the average.

### Transwell test

The transfected cells were inoculated into six-hole plates with 10^6^ cells/hole. When the fusion degree was 75%, the serum-free medium was replaced and cultured overnight. The cell density was adjusted to 10^5^ cells/ml. Ten microliters was taken and added to the upper chamber. Six hundred microliters of serum-containing medium was added to the lower chamber and cultured overnight. The chamber was removed and wiped off the cells in the upper chamber. After PBS washing, cells was fixed with methanol for 30 min, stained with 0.1% Crystal Violet for 20 min and washed with PBS. The cell invasion was observed under the microscope.

### Western blot detection

The transfected cells were collected. Lysates were added, and the cells were lysed on the ice for 30 min. Cells were centrifuged for 10 min (1000×***g***) to obtain supernatant, and then placed it in EP tube; 5× SDS sample loading buffer was added, and then boiled in boiling water for 10 min. After electrophoresis, the protein was transferred to PVDF membrane by using a membrane transfer instrument. Five percent skim milk was added to close the membrane for 2 h and washed off. Anti-I (1:1000) was added, and closed overnight at 4°C. The anti-I was removed by washing the film. HRP–conjugated goat anti-rabbit second antibody (1:5000) was added and exposed.

### Double fluorescein reporter enzyme

Luciferase reporter vector [psiCHECK2-LUCAT1- wild-type (WT), psiCHECK2-LUCAT1- Mutant (MUT)] and mimics-miR-199b-5p or miR-199b-5p-ininhibition were transfected into CC cells by liposomal method, respectively. After culturing for 5 h, fresh culture medium was replaced for continuous culture and transfected for 48 h.

#### Results

The binding force between miR-199b-5p and LUCAT1 was reflected by the ratio of the luminous intensity of sea cucumber luciferase and firefly luciferase.

### Co-immunoprecipitation detection

CC cells were lysed by using the EZMagna RIP kit and incubated with protein A magnetic beads, which was conjugated with an antibody at 4°C. After 6 h, the beads were washed with washing buffer and then incubated with 0.1 SDS/0.5 mg/ml protease K at 55°C for 30 min to remove proteins. Finally, the immunoprecipitation RNA was analyzed by qRT-PCR to prove the existence of LUCAT1 and miR-199b-5p by using specific primers.

### RNA pull-down experiment

CC cells were transfected with biotinylated miR-199b-5p-wt, miR-199b-5p-mut and negative control (GenePharma, Shanghai, China), respectively. After 48 h, the cell lysate was incubated with M-280 streptomycete magnetic beads (Invitgen) according to the production instructions. Then, qRT-PCR was applied to detect the level of LUCAT1 in the RNA complex binding to beads.

### Outcome measures

(1) The expression level of LUCAT1 in peripheral blood in the two groups; diagnostic value of LUCAT1 on CC; the connection between LUCAT1 and CC; the effect of LUCAT1 on the prognosis of CC patients. (2) Expression of LUCAT1 in CC cells; effect of LUCAT1 on biological behavior of CC cells. (3) Expression of miR-199b-5p in CC cells; effect of miR-199b-5p on biological behavior of CC cells. (4) The connection between LUCAT1 and miR-199b-5p in CC.

### Statistical methods

SPSS24.0 (Shanghai Yuchuang Network Technology Co., Ltd.) was used for statistical analysis of the experimental results. All the graphs results were drawn by using GraphPad8 (Shenzhen Tianruiqi Software Technology Co., Ltd.). The counting data were expressed as (%). The chi-square test was used for intergroup comparison. The measurement data were expressed as (mean number ± standard deviation). *t* test was used for intergroup comparison. One-way anova and LSD back-test were used for the comparison among groups. Repetitive measurement and analysis of variance and Bonferroni back-test were used to compare multiple time points. The diagnostic and predictive value was analyzed by ROC curve. The survival rate was calculated by Kaplan–Meier method. The comparison of survival rate was tested by log-rank test. The difference was statistically significant with *P*<0.050.

## Results

### Clinical significance of LUCAT1 on CC

Through detection, it could be concluded that the expression level of LUCAT1 in the peripheral blood and tissues of the patients in SG was higher than that in CG and adjacent tissues (*P*<0.050). According to ROC curve analysis, when the cut-off value was 1.635, the predictive sensitivity of LUCAT1 to CC was 67.16%, the specificity was 98.33%, the AUC was 0.808 and the 95% CI was 0.726–0.889, *P*<0.001. More details are shown in Figure 1.

**Figure 1:** Clinical significance of LUCAT1 on CC (**A**) LUCAT1 expression level in peripheral blood, *P<0.050. (**B**) LUCAT1 expression level in tissues, *P<0.050. (**C**) ROC curve of LUCAT1 for prediction of CC development.

### The connection between LUCAT1 and CC clinical pathology

After analysis, it could be concluded that LUCAT1 had no significant relationship with CC age, pathological changes and tissue types (*P*>0.050). However, it was closely related to CC differentiation, pathological stage and metastasis (*P*<0.001). More details are shown in Table 2.

**Table 2:** The connection between LUCAT1 and CC clinical pathology

	*n*	LUCAT1	*t* or F	*P*
Age (years)			0.242	0.809
≥55	39	1.94 ± 0.52		
<55	28	1.91 ± 0.47		
Pathological changes			0.047	0.986
Erosive type	26	1.89 ± 0.42		
Extrahepatic growing	20	1.94 ± 0.48		
Endophytic type	11	1.90 ± 0.50		
Ulcerative type	10	1.91 ± 0.46		
Histological types			0.119	0.949
Atypical hyperplasia	16	1.86 ± 0.40		
Carcinoma *in situ*	32	1.92 ± 0.36		
Invasive carcinoma	11	1.89 ± 0.38		
Adenocarcinoma	8	1.94 ± 0.42		
Differentiation			7.668	<0.001
Poorly differentiated	37	2.23 ± 0.28		
Middle+well differentiated	30	1.64 ± 0.35		
Pathological stage			4.942	<0.001
I–II	27	1.68 ± 0.34		
III–IV	40	2.16 ± 0.42		
Metastasis			5.055	<0.001
Yes	20	2.34 ± 0.46		
No	47	1.70 ± 0.48		

### Effect of LUCAT1 on prognosis of CC

The prognosis of CC patients was followed up for 3 years. Results: 62 patients were successfully followed up, with a follow-up success rate of 92.54%. Patients were divided into low LUCAT1 group (LUCAT1 < 1.92, *n*=27) and high LUCAT1 group (LUCAT1 ≥ 1.92, *n*=35) according to the median expression level of LUCA T1 in patients’ peripheral blood. The prognosis of the low LUCAT1 group was significantly better than that of the high LUCAT1 group by observing the 3-year survival in the two groups (*P*=0.030). More details are shown in Figure 2.

**Figure 2:** Survival curve of prognosis for 3 years

### Effect of LUCAT1 on CC cells

Detection of LUCAT1 expression level in C33A, HeLa, AV3 and H8 cells indicated that LUCAT1 expression level was higher in CC cells (*P*<0.050), with the highest expression level in C33A and AV3 (*P*<0.050). Therefore, C33A and AV3 were selected for subsequent experiments. After LUCAT1 was transfected into C33A and AV3, the biological behavior of cells was detected. It was found that the cell proliferation, invasion ability, Bcl-2 and Caspase-3 proteins in sh-LUCAT1 group were significantly higher than those in NC group and si-LUCAT1 group, while the apoptosis rate and Bax protein were significantly lower than those in NC group and si-LUCAT1 group (*P*<0.050). The proliferation ability, invasion ability, Bcl-2 and Caspase-3 proteins in si-LUCAT1 group were the lowest among the three groups, while the apoptosis rate and Bax protein were the highest among the three groups (*P*<0.050). More details are shown in Figure 3.

**Figure 3:** Effect of LUCAT1 on CC cells (**A**) Comparison of LUCAT1 expression levels in different CC cells, * represents comparison with C33A cells, *P*<0.050; ^#^ represents comparison with HeLa cells, *P*<0.050; ^@^ represents comparison with AV3 cells, *P*<0.050. (**B**) Proliferation of C33A cells after transfection with LUCAT1. (**C**) Proliferation of AV3 cells after transfection with LUCAT1. (**D**) Apoptosis rate and flow cytometry of C33A and AV3 cells after transfection with LUCAT1. (**E**) Invasion ability of C33A and AV3 cells after transfection with LUCAT1. (**F**) Protein expression and protein imprinting map of C33A cells after transfection with LUCAT1. (**G**) Protein expression and protein imprinting map of AV3 cells after transfection with LUCAT1.

### Effect of miR-199b-5p on CC cells

Detection of miR-199b-5p level in C33A, HeLa, AV3 and H8 cells indicated that miR-199b-5p was low expressed in CC cells (*P*<0.050). Since miR-199b-5p was transfected into C33A and AV3 cells, subsequent tests were carried out to detect their cell biological behaviors. It was found that the cell proliferation, invasion ability, Bcl-2 and Caspase-3 proteins of mimics-miR-199b-5p group were significantly lower than those of inhibition-miR-199b-5p group and NC-miR group, while the apoptosis rate and Bax protein were significantly higher than those of inhibition-miR-199b-5p group and NC-miR group (*P*<0.050). The proliferation ability, invasion ability, Bcl-2 and Caspase-3 proteins in NC-miR group were the lowest among the three groups, while the apoptosis rate and Bax protein were the highest among the three groups (*P*<0.050). The proliferation ability, invasion ability, Bcl-2 and Caspase-3 proteins in inhibition-miR-199b-5p group were the highest among the three groups, while the apoptosis rate and Bax protein were the highest among the three groups (*P*<0.050). More details are shown in Figure 4.

**Figure 4:** Effect of miR-199b-5p on CC cells (**A**) Comparison of miR-199b-5p expression levels in different CC cells, * represents comparison with C33A cells, *P*<0.050; ^#^ represents comparison with HeLa cells, *P*<0.050; *^@^* represents comparison with AV3 cells, *P*<0.050. (**B**) Proliferation of C33A cells after transfection with miR-199b-5p. (**C**) Proliferation of AV3 cells after transfection with miR-199b-5p. (**D**) Apoptosis rate and flow cytometry of C33A and AV3 cells after transfection with miR-199b-5p. (**E**) Invasion ability of C33A and AV3 cells after transfection with miR-199b-5p. (**F**) Protein expression and protein imprinting map of C33A cells after transfection with miR-199b-5p. (**G**) Protein expression and protein imprinting map of AV3 cells after transfection with miR-199b-5p.

### Connection between LUCAT1 and miR-199b-5p

Potential binding targets between LUCAT1 and miR-199b-5p were concluded by online target gene prediction of web analytics. The connection between LUCAT1 and miR-199b-5p was further verified by double fluorescein reporter enzyme, RIP and RNA pull-down experiments. The results indicated that the fluorescence activity of LUCAT1-WT was significantly inhibited by mimics-miR-199b-5p, while the levels of LUCAT1 and miR-199b-5p precipitated by Ago2 antibody were significantly higher than IgG. LUCAT1 was pulled down by biotin-labeled miR-199b-5p-WT, while miR-199b-5p-MUT could not pull down LUCAT1. Further, LUCAT1 and miR-199b-5p were co-transfected for biological function detection. The results indicated that the proliferation capacity of mimics-miR-199b-5p cells was correlated with mimics-miR-199b-5p transfection alone by up-regulation of LUCAT1 (sh-LUCAT1) and mimics-miR-199b-5p, and it was reversed (*P*<0.050), indicating that up-regulation of LUCAT1 could inhibit the expression of miR-199b-5p, promote the proliferation and invasion ability of CC cells and inhibit its apoptosis ability. More details are shown in Figure 5.

**Figure 5:** Connection between LUCAT1 and miR-199b-5p (**A**) Dual luciferase reporter enzyme; (**B**) RIP experiment; (**C**) RNA pull-down experiment; (**D**) proliferation of C33A cells; (**E**) proliferation of AV3 cells; (**F**) apoptosis rate; (**G**) cells invasion, *P<0.050.

## Discussion

CC, as the disease with the highest incidence among gynecologic malignant tumors, is a great threat worldwide [14]. Therefore, it is of great significance to fully understand the pathogenesis of CC for clinical prevention and treatment of CC. Recent studies have continuously confirmed the correlation between LncRNA and tumor diseases, which is currently a major research hotspot in clinical practice [15,16]. LncRNA is a long-chain non-coding RNA. In the study of Wei et al. [17], LncRNA XIST was found to be involved in the proliferation of pancreatic cancer, while Mao et al. [18] indicated that LncRNA LET promoted the invasion of migration of gastric cancer. LUCAT1, also known as SCAL1, is located on chromosome 5 and it was first found in respiratory epithelial cells of smokers. Current research is mostly limited to respiratory diseases and tumors [19,20]. However, this study is of great significance to clinical diagnosis and treatment of CC in the future by exploring the influence and mechanism of LUCAT1 on CC.

The results of this experiment indicated that LUCAT1 was highly expressed in the peripheral blood and tissues of CC patients, suggesting that LUCAT1 may be involved in the development and progression of CC. This was also the case when Zhou et al. [21] explored LUCAT1 in colorectal cancer, which also supported our experimental results. However, through ROC curve analysis, we found that the predictive sensitivity and specificity of detecting LUCAT1 in peripheral blood for CC occurrence were 67.16 and 98.33%, which had good diagnostic efficiency, suggesting that LUCAT1 could be used as a tumor marker for CC screening in future. Compared with traditional tumor markers such as CEA and CA125, LUCAT1 can make up for its deficiency in specificity, help clinical diagnosis of CC as early as possible and timely treatment and improve the prognosis of patients. In addition, we found that LUCAT1 was closely related to the differentiation, pathological stages and metastasis of CC by analyzing the relationship between LUCAT1 and CC’s clinical pathology, which further verified that LUCAT1 was involved in the progression of CC. We also found that LUCAT1 had certain influence on the prognosis of CC patients through prognosis follow-up, suggesting that LUCAT1 could not only be used as a clinical screening index for CC in the future, but also might be a potential therapeutic target for CC, which was of great significance for the prevention and treatment of CC. Therefore, in order to further understand the effect of LUCAT1 on CC, we transfected LUCAT1 into CC cells and detected its biological behavior. It was found that the proliferation, invasion ability and anti-apoptosis protein of CC cells were significantly reduced, while the apoptosis rate and apoptosis protein were significantly increased by inhibiting LUCAT1 expression, suggesting that LUCAT1 played a role of oncogenic gene in CC. This is also consistent with the results of Liu et al. [22] in exploring the influence mechanism of LUCAT1 on prostate cancer, which can support our experiment. At present, the pathway of LUCAT1 affecting CC is not clear. Looking up previous studies, we found that miR-199b-5p has abnormal expression in many tumor diseases [23,24], and it has been proved to have close relationship with CC [25]. Therefore, we detected the expression of miR-199b-5p in CC cells and found that it was low expression. We suspected that miR-199b-5p has a certain relationship with LUCAT1. In order to verify this point, we found that there was targeted binding between miR-199b-5p and LUCAT1 through double fluorescein reporter enzyme detection. Through RIP and RNA pull-down experiments, we found that the levels of LUCAT1 and miR-199b-5p precipitated by Ago2 antibody were significantly higher than IgG. RNA pull-down experiments found that LUCAT1 can be pulled down by biotin-labeled miR-199b-5p-WT, but cannot be pulled down by miR-199b-5p-MUT. The above experiments indicated that LUCAT1 could be used as ceRNA to regulate miR-199b-5p. However, transfection of LUCAT1 and miR-199b-5p into CC cells indicated that both up-regulation of miR-199b-5p and down-regulation of miR-199b-5p expression could increase the proliferation, invasion and decrease apoptosis of CC cells. This also confirmed that the expression changes of LUCAT1 and miR-199b-5p could cause changes in the biological behavior of CC cells. However, through co-transfection of sh-LUCAT1 and mimics-miR-199b-5p, we found that the proliferation and invasion ability of CC cells were inhibited and the significantly increased apoptosis ability was completely reversed after the original up-regulation of miR-199b-5p, which also confirmed that the targeted inhibition of miR-199b-5p by LUCAT1 promoted the development of CC. Looking up previous studies, we found that Kong et al. [26] proposed that LUCAT1 promotes the proliferation of oral cancer through PCNA, while Lou et al. [27] also confirmed that LUCAT1 promotes the occurrence of hepatocellular carcinoma by inhibiting ANXA2, which also confirmed that LUCAT1 has a consistent mechanism of action in a number of tumor diseases. Therefore, in-depth study of the impact of LUCAT1 may be a breakthrough for future CC and other tumor diseases.

To sum up, LUCAT1 was highly expressed in CC. It was involved in the tumor development of CC by targeting miR-199b-5p, which was of great significance for the diagnosis and treatment of CC in the future.

The present study was designed to explore the effect and mechanism of LUCAT1 on CC. However, due to the limited experimental conditions, there are still deficiencies. For example, data of benign CC patients are not collected in this experiment, so it is impossible to judge the specific role of LUCAT1 in benign CC lesions. In addition, due to the short experimental period, we do not yet know the impact of LUCAT1 on the long-term prognosis of CC patients. In this article, we suggested that LUCAT1 may be a potential therapeutic target for CC in the future, but we have not been able to carry out drug resistance and nude mice tumorigenesis experiments at this point, which is our research limitation. Moreover, the effect of LUCAT1 on CC is not only carried out by targeting miR-199b-5p. We do not yet know the signal pathway by which LUCAT1 targets miR-199b-5p to affect CC, which also needs more basic experiments to prove. We will conduct more in-depth, comprehensive and detailed experimental analysis for the above deficiencies as soon as possible, so as to obtain the best experimental results.

## Abbreviations

Ago2: argonaute2
AJCC: American Joint Committee on Cancer
BMI: BMI1 proto-oncogene
CC: cervical cancer
CCK-8: cell counting kit-8
CG: control group
EP: Eppendorf
LncRNA: long non-coding RNA
LUCAT1: lung cancer associated transcript 1
NC: negative control
RIPA: radioimmunoprecipitation assay buffer
ROC: receiver operating characteristic
SG: study group
TNM: tumor node metastasis
XIST: X inactive specific transcript
